The article "Activated α2-Macroglobulin Binding to Cell Surface GRP78 Induces T-Loop Phosphorylation of Akt1 by PDK1 in Association with Raptor" was retracted in 2025. Reasons: duplicated images; overlap with earlier publications; unreliable data; unreliable results or conclusions.

# Activated α_2_-Macroglobulin Binding to Cell Surface GRP78 Induces T-Loop Phosphorylation of Akt1 by PDK1 in Association with Raptor

**DOI:** 10.1371/journal.pone.0088373

**Published:** 2014-02-06

**Authors:** Uma Kant Misra, Salvatore Vincent Pizzo

**Affiliations:** Department of Pathology, Duke University Medical Center, Durham, North Carolina, United States of America; Florida International University, United States of America

## Abstract

PDK1 phosphorylates multiple substrates including Akt by PIP_3_-dependent mechanisms. In this report we provide evidence that in prostate cancer cells stimulated with activated α_2_-macroglobulin (α_2_M*) PDK1 phosphorylates Akt in the T-loop at Thr^308^ by using Raptor in the mTORC1 complex as a scaffold protein. First we demonstrate that PDK1, Raptor, and mTOR co-immunoprecipitate. Silencing the expression, not only of PDK1, but also Raptor by RNAi nearly abolished Akt phosphorylation at Akt^Thr308^ in Raptor-immunoprecipitates of α_2_M*-stimulated prostate cancer cells. Immunodepleting Raptor or PDK from cell lysates of cells treated with α_2_M* drastically reduced Akt phosphorylation at Thr^308^, which was recovered by adding the supernatant of Raptor- or PDK1-depleted cell lysates, respectively. Studies of insulin binding to its receptor on prostate cancer cells yielded similar results. We thus demonstrate that phosphorylating the T-loop Akt residue Thr^308^ by PDK1 requires Raptor of the mTORC1 complex as a platform or scaffold protein.

## Introduction

Tetrameric human α_2_-macroglobulin (α_2_M), a pan proteinase inhibitor, is expressed in most animal species [1]. The protein is synthesized by many cells and is present in plasma at a concentration of 1–5 µM. Tumors and their associated stroma also produce this protein as well as various proteinases that react with α_2_M [2]. When α_2_M reacts with a proteinase, the so called “bait region” in each subunit is cleaved followed by the rupture of a β-cysteinyl γ-glutamyl thiolester accompanied by a large conformational change in the molecule [3]. This exposes a receptor recognition site that is present in the carboxyl terminal domain of each subunit. Small nucleophiles such as methylamine or ammonia can directly rupture the thiolesters triggering a similar conformational change exposing the receptor recognition sites. These activated forms of α_2_M are designated α_2_M*. Although GRP78 (glucose regulated protein of M_r_ ∼78,000) is primarily known as a resident endoplasmic reticulum chaperone, it appears on the cell surface of many types of malignant cells [2], [4]–[9]. Binding of α_2_M* to tumor cell-surface GRP78 causes its autophosphorylation activating downstream pro-proliferative and anti-apoptotic signaling cascades including RAS/MAPK and PI 3-kinase/PDK1/Akt/mTORC1/mTORC2 [4]–[14].

The article "Activated α2-Macroglobulin Binding to Cell Surface GRP78 Induces T-Loop Phosphorylation of Akt1 by PDK1 in Association with Raptor" was retracted in 2025. Reasons: duplicated images; overlap with earlier publications; unreliable data; unreliable results or conclusions.

Activation of PI 3-kinase and subsequent production of PIP_3_ is the major signaling event triggered by cell binding of growth factors and hormones. Our previous studies suggest that α_2_M* functions like a growth factor triggering PI 3-kinase activation and production of PIP_3_ [2], [4]–[10], [13]. Most of the physiological effects of PIP_3_ in cells are mediated by AGC kinase family members that control cell proliferation, survival, and metabolic responses [15]–[19]. These include Akt (PKB) isoforms, S6-kinase (S6K), and PKC isoforms. PDK1 itself, a member of the AGC family, is the common upstream kinase phosphorylating and activating at least 23 AGC kinases [15]. AGC kinases have a common mechanism of activation which involves the dual phosphorylation of two residues lying within two highly conserved motifs, the T-loop (Thr^308^ for Akt1) and the hydrophobic motif (Ser^473^ for Akt1) [15]–[19]. Phosphorylation of both is required for full activation of Akt. Phosphorylation of Akt at Thr^308^ is indispensable for kinase activity whereas phosphorylation of Ser^473^ enhances kinase activity by fivefold [20]. In the case of Akt, conformational change induced by PIP_3_ binding to its PH domain promotes its phosphorylation by PDK1. PDK1 localizes at the plasma membrane through its COOH-terminal pH domain which binds to PIP_3_ and facilitates the colocalization of Akt and PDK1 [15]–[19]. In PDK1 mutants that cannot bind PIP_3_, Akt is not phosphorylated at Thr^308^ [21], [22]. Thus other mechanisms might operate to enable Akt and PDK1 to interact at the membrane including PDK1 binding to scaffolding components such as growth factor receptor-bound protein 14 (GRB14) [23] or five repressor element under dual repression binding protein1 (FREUD1) [24]. Lys^63^ linked ubiquitylation of Akt by the TNF receptor-associated factor (TRAF6) ligase also facilitates its recruitment to the plasma membrane [25]. The cellular distribution of PDK1 is dependent on distinct mechanisms including binding to soluble inositol phosphates that cause PDK1 localization in the cytosol, where many of its non-phosphoinositide-binding substrates reside [26]. PDK1 also binds to mAKAPα forming a complex with ERK and RSK, which enables RSK activation [27]. PDK1 is observed in the nucleus as well as in the cytoplasm [28].

Other mechanistic studies have probed the role of the PIF-pocket in PDK1 activity. Activation of AGC kinases that do not possess a PH domain is triggered through phosphorylation of their hydrophobic (HF) motif by mTORC1, which promotes that interaction with a motif in the PDK1 catalytic domain [15]–[19]. PDK1 then phosphorylates the T-loop residues eliciting activation. Mutation of the PIF-pocket abolished activation of S6K and SGK1 isoforms but does not affect PDK1-mediated Akt^308^ phosphorylation [15]–[19]. *In vitro* studies using mutation of Ser^473^ to alanine has no effect on phosphorylation of Akt^Thr308^ and activation of Akt [29]. The PDK1 inhibitor GSK2334470 inhibited T-loop phosphorylation of S6K and SGK, but was ineffective at suppressing Akt^308^ phosphorylation and hence Akt activation [30].

mTOR plays an important role in cell metabolism, proliferation, differentiation, and survival [31]–[35]. mTOR contains multiple HEAT repeats at the amino terminal half and a serine-threonine kinase domain in the carboxyl-terminal region, flanked by regulatory FAT and FATC regions. This structure provides the binding sites for multiple proteins that interact with mTOR, regulating its activity and subcellular localization. Scaffold proteins co-localize the molecules involved in the same signaling pathways and function as catalysts thereby activating different components in the signaling pathways [36]. Post-translational modifications resulting from the activity of a kinase can facilitate interactions of the targeted molecule(s) with other proteins which enable to simultaneously localize two or more other proteins. Scaffold proteins are instrumental in ensuring specificity and efficiency in regulating positive and negative feedback loops [37]. Activation of Akt via mTORC signaling is scaffold-dependent [38]. The catalytically active mTOR subunit exists in two independent multiprotein complexes, mTORC1 and mTORC2, with different regulatory properties and cellular activities. Assembly of these complexes is regulated by mTOR interacting proteins [34], [35]. Some proteins interact constitutively with mTOR complexes, while others are transient partners regulated by phosphorylation or other factors [37], [38]. The identity of mTORC1 and mTORC2 is defined by whether Raptor or Rictor, respectively are part of the complex. Raptor contains three HEAT repeats at the amino terminal domain and seven WD40 repeats in the carboxyl-terminal domain that recruit mTORC1 substrates [39].

The article "Activated α2-Macroglobulin Binding to Cell Surface GRP78 Induces T-Loop Phosphorylation of Akt1 by PDK1 in Association with Raptor" was retracted in 2025. Reasons: duplicated images; overlap with earlier publications; unreliable data; unreliable results or conclusions.

Recruiting PDK1 to muscle A kinase anchoring protein (mAKABα) facilitates activation and release of the downstream target RSK [36]. Functions of PDK1 are also regulated by changes in its conformation, protein-protein interaction, and its subcellular localization [15]–[19]. Several proteins interact with PDK1 modulating its activity and subcellular localization as already noted above [27], [36], [40]–[43]. In addition to its function as a master kinase in receptor tyrosine kinase signaling, PDK1 functions as an adaptor protein in several signaling events independent of its kinase activity such as enhancing the GEF activity of RalGDS [44] and T-cell development by activating PKC and also acting as an adaptor in recruiting PKC and CARD11 to regulate IKK and NFκB [45]. Thus PDK1 may function in more diverse signaling pathways as a kinase, as a scaffold protein, and/or a kinase-independent regulatory protein. AKT is predominantly localized in cytoplasm and the ER [46]. On growth factor stimulation a substantial translocation of Akt to the plasma membrane occurs. Recently studies demonstrate that mTORC2-dependent phosphorylation of Akt on Ser^473^ takes place on the surface of the ER [46]. Phosphorylation of Akt at Thr^308^ and Ser^473^ have been reported as either interdependent or independent of each other [46], but in either case both PDK1 and mTORC2 must be in close spatial proximity for efficient phosphorylation of Akt at both Thr^308^ and Ser^473^, respectively. Here we hypothesize that Raptor interacts physically with PDK1 in the mTORC1 signaling complex serving as a scaffolding protein which allows PDK1 to phosphorylate Akt at Thr^308^. We show that PDK1 co-immunoprecipitates with Raptor, and mTOR in α_2_M*-stimulated prostate cancer cells. Downregulation of Raptor or PDK1 by RNAi nearly abolishes α_2_M* -induced phosphorylation of Akt at Thr^308^. Immunodepletion of PDK1 or Raptor reduced Akt at Thr^308^ significantly. Addition of the supernatant of Raptor or PDK1 depleted cell lysates restored Akt^Thr308^ phosphorylation. Thus, PIP_3_ production is a necessary, but not sufficient event in activating Akt by phosphorylation at Thr^308^. Whether these results will apply to activation of other PH domain-containing AGC kinases by PDK1 remains to be determined, but seems likely.

## Materials and Methods

### Materials

Culture media were purchased from Invitrogen. Activated α_2_-macroglobulin (α_2_M*) was prepared as described previously [2]. Antibodies against mTOR, p-Akt^Thr308^, p-Akt^Ser473^, Akt, and PDK1 were purchased from Cell Signaling Technology (Danvers, MA). Antibodies against Raptor were purchased from Santa Cruz Biotechnology (Santa Cruz, CA). Anti-actin antibody was from Sigma (St. Louis, MO). [^33^P]-γ-ATP (specific antibody 3000 Ci/mmol) was purchased from Perkin-Elmer Life Sciences (Waltham, MA). All other materials were of analytical grade and procured locally.

### Prostate cancer cell lines

We have used two human prostate cancer cell lines 1-LN and DU-145. The highly metastatic 1-LN cell line is derived from less metastatic PC-3 cells in nude mice and was a kind gift of Dr. Philip Walther (Duke University Medical Center, Durham, NC) [12]. DU-145 cells were purchased from ATCC (Manassas, VA). Cells were grown in 6 or 12 well plates in RPMI 1640 medium supplemented with 10% FBS 2 mM glutamine, 12.5 units/ml penicillin, 6.5 µg/ml streptomycin and 10 nM insulin (RPMI-S), in a humidified CO_2_ incubator at 37°C. After reaching 90% confluency, the medium was aspirated and a fresh volume of RPMI-S medium and the cells were used for experiments described below.

The article "Activated α2-Macroglobulin Binding to Cell Surface GRP78 Induces T-Loop Phosphorylation of Akt1 by PDK1 in Association with Raptor" was retracted in 2025. Reasons: duplicated images; overlap with earlier publications; unreliable data; unreliable results or conclusions.

### Co-immunoprecipitation of PDK1 with Raptor and mTOR in prostate cancer cells stimulated with α_2_M*

Colocalization of interacting proteins has been widely studied by co-immunoprecipitation techniques. To test the hypothesis PDK1 is an interacting protein with Raptor in the mTOR signalosome, we first studied the colocalization of PDK1 with mTOR, and Raptor by co-immunoprecipitation in α_2_M*-stimulated cells. 1-LN cells were grown over night in RPMI-S media in 6 well plates (3×10^6^ cells/well) at 37°C in a humidified CO_2_ (5%) incubator. At about 90% confluency the medium was aspirated, cells washed 2x with cold HHBSS, a volume of RPMPI-S added and after 5 min of temperature equilibration; cells in respective were stimulated with either buffer or α_2_M* (50 pM/25 min) and incubated as above. The reaction was terminated by aspirating the media, and cells lysed in a volume of CHAPS lysis buffer B containing 40 mM HEPES (pH 7.5, 120 mM NaCl, 1 mM EDTA, 10 mM sodium pyrophosphate, 10 mM β-glycerophosphate, 0.5 mM sodium orthovanadate, 0.3%, CHAPS and a Roche protease inhibitor cocktail tablet (1 tablet/10 ml) was added and cells lysed over ice for 15 min. The lysates were transferred to separate Eppendorf tubes, centrifuged (1000 rpm/5 min/4°C) and supernatants used for protein estimation and immunoprecipitation. Equal amounts of lysate proteins (200–250 µg) in separate experiments were used for immunoprecipitation with Raptor antibodies (1∶50, Santa Cruz Cat # SC81537). PDK1 antibodies (1∶50) and mTOR antibodies (1∶50) followed by the addition of 40 µl protein A agarose and contents incubated with rotation overnight at 4°C. Raptor, PDK1, mTOR immunoprecipitates were recovered by micro-centrifugation (2000 rpm/5 min/4°C) and washed twice with cold lysis buffer B. To each immunoprecipitate a volume of 4x sample buffer was added, tubes boiled for 5 min centrifuged, electrophoresed (4–20% or 10% acrylamide gels), transferred to Hybond-P membranes and the respective membranes immunoblotted with Raptor, PDK1, and mTOR antibodies. The protein bands on the membranes were visualized by ECF and STORM 860 Phosphorimager (GE Lifesciences). The specificity of antibodies employed here and in the experiments described below was determined by treating the cells with non-immunoantibodies and cell lysates processed as above under the experimental conditions, no reactivity of these controls was observed. The membranes were reprobed for protein-loading controls [12], [47]. Total cell lysates of cells treated as above were also immunoblotted for mTOR, Raptor, and PDK1 like in their immunoprecipitates.

The article "Activated α2-Macroglobulin Binding to Cell Surface GRP78 Induces T-Loop Phosphorylation of Akt1 by PDK1 in Association with Raptor" was retracted in 2025. Reasons: duplicated images; overlap with earlier publications; unreliable data; unreliable results or conclusions.

### Silencing expression of PDK1 and Raptor genes by RNAi

To understand the mechanistic details of phosphorylation of Akt at Thr^308^ by PDK1, we have used RNAis to downregulate the expression of PDK1 or Raptor. The chemical synthesis purification and annealing of PDK1 dsRNA were performed by Ambione of Raptor by Sigma. The PDK1 sense sequence is 5′ - CAG AAG AUC AUU AAG UUG CAA-3′; antisense 5′ - UUA CAA CUU AAU GAU CUU CUG-3′. The Raptor sense sequence is: 5′ - CUC AAC AAA UCU UUG CAG At-3′ (ID# SAS1_HSO1_00048387); antisense 5′ - UCU GCA AAG AUU UGU UGA Gels - 3′ (ID# SAS1_Hs) 1-00048387_AS.

### The effect of silencing PDK1 or Raptor gene expression by RNAi on p-Akt^Thr308^ phosphorylation in prostate cancer cells stimulated with α_2_M*

In all the experiments described below, downregulation of PDK1 or Raptor expression was achieved by transfecting the cancer cells with the respective dsRNAs (100 nM/48 h). Downregulation of PDK1 or Raptor, as measured by Western blotting, was ∼65–70% [12]. Prostate cancer cells grown overnight (1×10^6^ cells/well 6 well plates) were treated as follows: (1) lipofectamine + buffer; (2) lipofectamine + α_2_M* (50 pM/25 min); (3) respective dsRNA (100 nM/48 h) then α_2_M* (50 pm/25 min); or (4) scrambled dsRNA (100 nM/48 h) then α_2_M*. We have used insulin (200 nM/15 min) as a positive control in these studies. The reactions were terminated by aspirating the medium, a volume of CHAPS lysis buffer added, cells lysed over ice for 15 min, centrifuged (1000 pm/5 min/4°C), supernatants transferred to new tubes and protein concentration determined. As desired, equal amounts of lysate proteins (200–250 µg) were immunoprecipitated with either anti-PDK1 or Raptor antibodies as described above. Phosphorylation of Akt at Thr^308^ by PDK1 or Raptor immunoprecipitates was determined by kinase assays described elsewhere [2], [6], [7], [9], [12], [47]. Briefly, the respective immunoprecipitates were washed with CHAPS lysis buffer B, supplemented with 0.5 M NaCl; lysis buffer B and Tri•HCl (pH 7.4) supplemented with 1 mM DTT, 1 mM PMSF and 1 mM benzamidine by centrifugation at 2,500 rpm for 5 min at 4°C. To each immunoprecipitate 40 µl of kinase buffer containing 50 mM Tris•HCl (pH 7.5) 10 mM Mg Cl_2_, 1 mM DTT, 1 mM PMSF, 1 mM benzamidine and 20 µg/ml leupeptin was added followed by the addition of 30 µM Akt^Thr308^ kinase substrate (NH_2_-KTFCGTPEYLAPEVRR-COOH) to the respective tubes. The peptide (NH_2_- GGEEEELYFELVKKKK-COOH (ZAK2 peptide) served as the control. The reaction was initiated by adding 50 µM ATP and 5 µCi [^33^P]-γ-ATP in each tube and tubes incubated for 30 min at 30° in a shaking water bath. The reaction was stopped by the addition of 5 µl of 0.5 M EDTA in each tube. The tubes centrifuged at 3000 rpm for 3 min, 40 µl of each supernatant applied on p81 phosphocellulose paper, allowed to dry and paper washed four times each time by immersing them in a liter of 1N H_3_PO_4_ for 3 min. The papers were rinsed with acetone and that radioactivity was counted in a liquid scintillation counter. In preliminary experiments kinase activities of Akt^Thr308^ kinase towards ZAK3 peptide were always 50 to 60% of buffer control. Hence control peptide activities are not being shown.

The article "Activated α2-Macroglobulin Binding to Cell Surface GRP78 Induces T-Loop Phosphorylation of Akt1 by PDK1 in Association with Raptor" was retracted in 2025. Reasons: duplicated images; overlap with earlier publications; unreliable data; unreliable results or conclusions.

### Determination of the effect of immunodepletion of Raptor and PDK1 in cell lysates of stimulated cells on Akt^Thr308^ phosphorylation

In addition to down regulating the expression of Raptor and PDK1 respective by RNAis on α_2_M/insulin stimulated Akt^Thr308^ phosphorylation by PDK1, we also studied the effect of immunodepleting Raptor and PDK1 on Akt^Thr308^ phosphorylation. The 1-LN prostate cancer cells were grown and stimulated with α_2_M* (50 pM/25 min) or insulin (200 nM/15 min) as described above. The reaction was terminated by expirating the media and cells lysed in lysis buffer A containing 50 mM Tris•HCl (pH 7.5) 120 mM NaCl 0.1% NP40, 25 mM sodium fluoride, 1 mM sodium pyrophosphate, 0.1 mM sodium orthovanadate, 1 mM PMSF, 1 mM benzamidine and leupeptin (10 µg/ml) as above. The lysates were centrifugated at 1000 rpm/5 min/4°C, supernatants collected and protein concentration determined. In separate experiments to deplete PDK1 and Raptor in cell lysates, to an equal amount of lysate protein was added anti-PDK1 or Raptor antibody and immunoprecipitation of PDK1 and Raptor was done as described above. Washed PDK1 and Raptor immunoprecipitates were used for the assay of Akt^Thr308^ phosphorylation in absence or presence of cell lysates remaining after removal of PDK1 or Raptor, which was assessed by immunoblotting of PDK1 and Raptor and found to be negligible (data not shown). Akt^Thr308^ phosphorylation was assayed as described above.

### Statistical analysis

Statistical analysis significance of the data was determined by students “t” test. P values of 0.05 are considered statistically significant.

## Results

### Raptor and PDK1 co-immunoprecipitate

Stimulation of 1-LN prostate cancer cells with α_2_M* causes a 2-3-fold increase in mTOR, Raptor, p-S6K, P-4EBP1, p-Akt^Thr308^, and p-Akt^Ser473^ in a time and dose-dependent manner [12]. To examine the interaction and co-localization of PDK1 and Raptor in the current study, we first performed co-immunoprecipitation studies. 1-LN cells stimulated with α_2_M* demonstrated co-immunoprecipitation of mTOR, Raptor, and PDK1 (Figure 1). These studies suggest interaction between mTOR or Raptor may facilitate PDK1-dependent downstream signaling induced in prostate cancer cells stimulated with α_2_M*. Since Raptor is a scaffold protein and does not have a kinase function, we suggest that PDK1 uses Raptor as a platform for phosphorylating Akt at Thr^308^.

The article "Activated α2-Macroglobulin Binding to Cell Surface GRP78 Induces T-Loop Phosphorylation of Akt1 by PDK1 in Association with Raptor" was retracted in 2025. Reasons: duplicated images; overlap with earlier publications; unreliable data; unreliable results or conclusions.

**Figure 1:** Effect of α_2_M* treatment of 1-LN cancer cells on Raptor interaction with PDK1. **Panel A**. Co-immunoprecipitation of mTOR, Raptor, and PDK1 in 1-LN prostate cancer cells stimulated with α_2_M* (50 pM/20 min/37°C). The lanes in immunoblots are: (1) buffer control and (2) α_2_M* stimulated. A representative immunoblot of three to four independent experiments is shown. **Panel B**. Representative immunoblots of mTOR, Raptor, and PDK1 in cell lysates of 1-LN prostate cancer cells stimulated with α_2_M* (50 pM/20 min/37°C) from three to four experiments along with the protein loading control actin.

### Inhibition of α_2_M*-induced Akt^Thr308^ phosphorylation Raptor immunoprecipitates of prostate cancer cells transfected with dsRNA of PDK1 and Raptor, respectively

To further probe the proposed interaction of Raptor with PDK1 in the phosphorylation of Akt at Thr^308^ we silenced the expression of PDK1 or Raptor by RNAi and obtained Raptor immunoprecipitates from cells stimulated with α_2_M* (Figure 2). In prostate cancer cells transfected with PDK1 dsRNAi, PDK1 was reduced ∼65–70% (Figure 2A) and in cells transfected with Raptor dsRNA levels of Raptor were reduced by about the same degree [12]. As expected, in prostate cancer cells stimulated with α_2_M*, silencing PDK1 gene expression significantly reduced phosphorylation of Akt at Thr^308^ as determined by Western blotting to detect p-Akt^Thr308^ in cell lysates (Figure 2B). These studies demonstrate that PDK1 is the Akt^Thr308^ kinase. We have shown earlier that down regulation of Raptor by RNAi significantly reduced phosphorylation of S6K at Thr^389^ and Thr^229^ and 4EBP1 [12]. S6K and 4EBP1 are direct down stream targets of mTORC1 which phosphorylates S6K at Thr^389^ while PDK1 phosphorylates S6K at Thr^229^. Since down regulation of Raptor not only reduced phosphorylation of S6K at Thr^389^ mediated by mTORC [12], but also phosphorylation of S6K at Thr^229^ we suggest that Raptor plays a role in the kinase activity of PDK1. We thus next studied phosphorylation of Akt at Thr^308^ by PDK1 employing kinase assays in Raptor immunoprecipitates of cells transfected Raptor RNAi and stimulated with α_2_M* (Figure 2A). Silencing Raptor gene expression nearly abolished α_2_M*-induced phosphorylation of Akt at Thr^308^ (Figure 2). Thus co-immunoprecipitation studies (Figure 1) and Raptor RNAi studies show that Raptor and PDK1 are interacting proteins in the phosphorylation of Akt at Thr^308^ and deficiency of either suppresses phosphorylation of Akt at Thr^308^. Similar results were obtained on phosphorylation of Akt at Thr^308^ in Raptor and PDK1 immunoprecipitates of 1-LN and DU-145 prostate cancer cells transfected with PDK1 and Raptor dsRNAs (Figure 3). Insulin has been widely used to study mTOR signaling. We also compared the effect of down regulating PDK1 expression by RNAi on Akt^Thr308^ phosphorylation in Raptor immunoprecipitates of 1-LN cells stimulated with insulin as well as α_2_M* (Figure 4). We show that stimulation of cells with insulin yielded comparable results. Prolonged activation of mTORC1 causes feedback inhibition of PI 3-kinase/Akt signaling. However, in this study we employed 20 min incubation in all experiments. In this short time period it is unlikely that feedback inhibition of PI 3-kinase/Akt signaling would occur and affect Akt^T308^ phosphorylation by PDK1. Since Raptor does not possess kinase activity, Raptor and PDK1 immunoprecipitates of cell lysates should demonstrate the same ability to phosphorylate Akt at Thr^308^ as is found in the current study. These studies further support our hypothesis that Raptor in the mTORC1 complex is required for PDK1-mediated T-loop phosphorylation of Akt and suggest that like mTORC2, mTORC1 complex also participates in Akt activation.

The article "Activated α2-Macroglobulin Binding to Cell Surface GRP78 Induces T-Loop Phosphorylation of Akt1 by PDK1 in Association with Raptor" was retracted in 2025. Reasons: duplicated images; overlap with earlier publications; unreliable data; unreliable results or conclusions.

**Figure 2:** PDK1 co-immunoprecipitates with Raptor. Bar diagram showing the presence of PDK1 in cell lysates (**Panel A**) and p-Akt^Thr308^ in Raptor immunoprecipitates (**Panel B**) from 1-LN and DU-145 cells transfected with PDK1 dsRNA and stimulated with α_2_M* (50 pM/20 min/37°C). A representative immunoblot of PDK1 and p-Akt^Thr308^ from triplicate experiments is shown below the respective bar diagrams. The lanes in the bar diagram and immunoblots of PDK1 and p-Akt^Thr308^ are: (1) lipofectamine + buffer; (2) lipofectamine and α_2_M*; (3) dsPDK1 RNAi (100 nM/48 h/37°C) then α_2_M*; and (4) scrambled dsRNAi (100 nM/48 h/37°C) then α_2_M*. PDK1 protein is expressed as the ratio of PDK1/actin and that of p-Akt^Thr308^ in arbitrary fluorescent units (x10^3^). Values significantly different from transfected cells at 5% levels are marked with an asterick (*). **Panel C.** Representative immunoblots from three experiments of p-Akt^Thr308^ and p-Akt^Ser473^ in Raptor immunoprecipiates of 1-LN cells stimulated with α_2_M*. The lanes in immunoblots are: (1) buffer; (2) α_2_M* (50 pM/20 min/37°C).

**Figure 3:** T-loop phosphorylation of Akt at Thr^308^ in Raptor or PDK1 immunoprecipitates of 1-LN or DU-145 cells transfected with dsPDK1 or dsRaptor-RNAi, and stimulated with α_2_M*. The T-loop phosphorylation was determined by kinase assay. The bars in the diagram are: (1) lipofectamine + buffer; (2) lipofectamine + α_2_M* (50 pM/20 min); (3) lipofectamine + dsRaptor RNAi (100 nM/48 h) or dsPDK1 RNAi (100 nM/48 h) then α_2_M*; and (4) scrambled dsRNA (100 nM/48 h) then α_2_M*. The Akt phosphorylation is expresed as fmol [^33^P]-γ-ATP incorporated/mg cell protein and is mean ± SE from three to four independent expermients in each case.

**Figure 4:** Suppression of α_2_M* or insulin-induced phosphorylation of Akt at Thr^308^ in Raptor immunoprecipitates of 1-LN cells transfected with dsPDK1 RNAi. The bars in the diagram are: (1) lipofectamine + buffer; (2) lipofectamine + α_2_M* (50 pM/20 min); (3) dsPDK1 RNA (100 nM/48 h) then α_2_M*; (4) lipofectamine + insulin (200 nM/20 min); (5) dsPDK1 RNAi (100 nM/20 min) then α_2_M*; (5) dsPDK1 RNAi (100 nM/20 min) then insulin (200 nM/20 min); (6) scrambled dsRNAi (100 nM/48 h) then insulin (200 nM/20 min). The phosphorylation is expressed as fmol [^33^P]-γ-ATP incorporated/mg protein) and is mean ± SE from three independent experiments in each case.

### Suppression of phosphorylation of Akt at Thr^308^ in prostate cancer cells stimulated with α_2_M* and cell lysates immunodepleted of Raptor or PDK1, respectively

To further analyze the requirement of Raptor in Akt phosphorylation at Thr^308^ by PDK1, we immunodepleted α_2_M*-stimulated 1-LN cell lysates of Raptor with anti-Raptor or PDK1 antibodies. We measured phosphorylation of Akt at Thr^308^ by kinase assay in Raptor or PDK1 immunoprecipitate in absence or in presence of cell lysates depleted of Raptor (Figure 5A) or PDK1 of cells stimulated with α_2_M* or insulin (Figure 5B). Raptor immunoprecipitates in the absence of Raptor depleted lysates showed little or negligible Akt phosphorylation at Thr^308^ in both α_2_M and insulin-stimulated cells (Figure 5A and B). Addition of Raptor-depleted lysates to the reaction mixture resulted in several fold increase in Akt^Thr308^ phosphorylation (Figure 5A). This is largely because of PDK1 remaining in the Raptor-depleted cell lysates. Similar results were obtained in cells depleted of PDK1. Immunoprecipitates of PDK1 in the absence of PDK1 depleted cell lysates showed little or negligible phosphorylation of Akt^Thr308^ in both α_2_M* and insulin-stimulated cells (Figure 3B). Addition of PDK1-depleted cell lysates resulted in a several fold increase in phosphorylation of Akt at 308 (Figure 5B). These results demonstrate the requirement of Raptor for phosphorylation of Akt at Thr^308^ by PDK1 and indicate the assembly of multiprotein signaling complex in initiating PDK1 signaling network. Formation of a similar multiprotein signaling complex has recently been suggested.

The article "Activated α2-Macroglobulin Binding to Cell Surface GRP78 Induces T-Loop Phosphorylation of Akt1 by PDK1 in Association with Raptor" was retracted in 2025. Reasons: duplicated images; overlap with earlier publications; unreliable data; unreliable results or conclusions.

**Figure 5:** Raptor immunodepletion and Akt^Thr308^ phosphorylation. **Panel A**. Effect of immunodepletion of Raptor in cell lysates of 1-LN cells stimulated with α_2_M* (50 pM/20 min) or insulin (200 nM/20 min) on Akt^Thr308^ phosphorylation. **Panel B**. Same as in **Panel A** except in cell lysates PDK1 was immunodepleted. Phosphorylation of Akt at Thr^308^ in **Panels A and B** was determined by kinase assay in Raptor immunoprecipitates from cells stimulated with: (1) buffer; (2) α_2_M* or insulin; and (3) α_2_M* or insulin + cell lysates of Raptor (**Panel A**) or PDK1 depleted cells (**Panel B**). Phosphorylation of Akt at Thr^308^ is expressed as fmol [^33^P]-γ-ATP/mg cell protein and is the mean ± SE from three independent experiments.

## Discussion

PDK1 is a serine/threonine kinase that phosphorylates members of the conserved AGC kinase family including Akt at Thr^308^ and is implicated in critical cellular processes including survival, metabolism, and tumorigenesis. Activation of PDK1 in cancer through genomic or epigenetic changes is often associated with more aggressive tumors and poor prognosis.

Activated α_2_M* binds to cell surface GRP78 and activates downstream pro-proliferative and anti-apoptosis signaling cascades including RAS/MAPK, PI 3-kinase, PDK1, Akt and mTORC1 and mTORC2 signaling [4]–[14]. Raptor is an essential component of the mTORC1 complex which regulates mTORC1 activity [34], [35]. Mice deficient in either Raptor or mTOR show serious developmental abnormalities [48]–[50]. For example, Raptor deficient mice become progressively dystrophic, tissues are impaired in their oxidative capacity, and cells contain increased glycogen stores [51], [53]. Silencing Raptor or mTOR expression by RNAi equally decreases phosphorylation of S6K and 4EBP1, the direct downstream targets of mTORC1 [54]. Actively dividing cells transfected with Raptor RNAi show reductions in cell size and decreased S6K phosphorylation [54]. Since Raptor is without any enzyme activity, Raptor appears to modulate mTORC1 function by serving as a platform for mTORC1 activity. The assembly of proteins into multiprotein complexes is an important mechanism that allows cells to carryout diverse functions that the individual proteins of the complex could not perform on their own. Using co-immunoprecipitation techniques it has been shown that Raptor forms a multiprotein complex of 4EBP1, S6K, mTOR, HERT, Akt and HSP90 in DU-145 cells and thereby it regulates telomerase activity [55]. Akt co-exists with ERK1/2 in a multiprotein complex containing PDK1 and RSK in MK-PT cells [56]. TFII-I also is a binding partner of Akt in Neuro 2A cells [57]. PDK1 is upstream of mTORC1-Raptor. PDK1 plays important role in the regulation of cellular responses in multiple organs by mediating PI 3-kinase signaling pathways through activating AGC kinases [15]–[19]. PDK1-mediated phosphorylation of Akt at Thr^308^ does not occur in either PDK1 null mice embryonic stem cells or tissue specific PDK1-knockdown mice [17], [26], [50]. Knockdown of PDK1 in pancreatic β cell in mice results in progressive hyperglycemia [52]. In endothelial cell like Raptor, PDK1 maintains glucose homeostasis. Like Raptor, PDK1 knockout mice are embryonic lethal. Knock-in mice expressing a mutant of PDK1 incapable of binding to phosphoinositide were significantly smaller, insulin resistant, and hyperglycemic. Phosphorylation of Akt at Thr^308^ in these mice was markedly reduced [22]. The cellular responses elicited in Raptor and PDK1 deficient mice are quite similar. PDK1 is upstream of Raptor-mTORC1, therefore it is very likely Raptor plays an important role in PDK1-mediated signaling network.

The article "Activated α2-Macroglobulin Binding to Cell Surface GRP78 Induces T-Loop Phosphorylation of Akt1 by PDK1 in Association with Raptor" was retracted in 2025. Reasons: duplicated images; overlap with earlier publications; unreliable data; unreliable results or conclusions.

Regulation of PDK1 activity occurs by several mechanisms including post-translational phosphorylation, which induces conformational changes stabilizing the protein, serving as anchors with respect to interaction with other proteins, or regulating the intracellular targeting of PDK1 to specific compartments such as cytoplasm, plasma membrane or the nucleus [15]–[19]. PDK1 is constitutively active. However, PDK1 is activated in membrane rafts in response to growth factors [58]. PDK1 exists as a dimer in cells and phosphorylation of the pH domain residue Thr^513^ regulates PH domain dimer-monomer equilibrium thereby converting an inactive dimer to an active monomer. Membrane bound PDK1, self-activates via autophosphorylation resulting in phosphorylation of the activation loop residue Ser^241^ and of PH domain residues Ser^410^ and Thr^513^. Subsequently, the active PDK1 kinase can phosphoactivate plasma membrane targets or can dissociate from membrane and phosphorylate cytoplasmic targets [59]. Dimerization of PDK1 may be due to the differential regulation of various pools of cytosolic PDK1. It is likely that active PDK1 monomers which dissociated from the plasma membrane may bind to Raptor and phosphorylate Akt at Thr^308^ [60]. Polyphosphoinositide PI (3,5) P2 is required for full activation and localization of mTORC1 by insulin and amino acids due to its interaction with WD40 domain of Raptor [61].

The article "Activated α2-Macroglobulin Binding to Cell Surface GRP78 Induces T-Loop Phosphorylation of Akt1 by PDK1 in Association with Raptor" was retracted in 2025. Reasons: duplicated images; overlap with earlier publications; unreliable data; unreliable results or conclusions.

The PI 3-kinase inhibitor LY294002, inhibits phosphorylation of Akt at Thr^308^ in mTOR immunoprecipitates of prostate cancer cells stimulated with α_2_M* [12]. Akt^Thr308^ phosphorylation, therefore, is PIP_3_-dependent and should take place at the plasma membrane. We do not understand the precise mechanistic and subcellular location of Raptor-mediated phosphorylation of Akt at Thr^308^ reported here. PDK1 in unstimulated cells is mostly cytosolic in occurrence, but stimulation with growth factors causes translocates to plasma membranes. PDK1 also may translocate to nuclei [62]. Akt is predominantly located in the cytoplasm and ER. After growth factor stimulation, a substantial translocation of Akt occurs. mTOR and Raptor are predominantly located in the ER and Golgi [63], [64]. Recently studies demonstrate that mTORC2-dependent phosphorylation of Akt^S473^ occurs on the surface of the ER [64]. Phosphorylation of Akt at Thr^308^ and Ser^473^ have been reported to be both interdependent or independent of each other [46], but in either case both PDK1 and mTORC2 must be in close spatial proximity for efficient phosphorylation of Akt at both Thr^308^ and Ser^473^, respectively. This view is substantiated by the presence of both p-Akt^Thr308^ and p-Akt^Ser473^ in Raptor immunoprecipitates of 1-LN cells stimulated with α_2_M* (Figure 3). We have recently demonstrated that in prostate cancer cells treated with a cAMP analogue, Raptor is a co-factor for PDK1-dependent phosphorylation of Akt at Thr^308^ [65]. In this previous report, however, we did not study cell surface ligation by a characterized ligand to determine whether in receptor-mediated activation of the PI 3-kinase/Akt/mTOR pathway, Raptor performs such a function.

In conclusion, in this study we employ co-immunoprecipitation, RNAi, and immunodepletion techniques to demonstrate that PDK1-mediated phosphorylation of Akt^Thr308^ requires Raptor as a scaffold or co-factor in addition to the requirement for phosphoinositide participation in Akt activation. Thus PIP_3_ generation is a necessary, but not sufficient requirement in PDK1-dependent phosphorylation of Akt^Thr308^. A recent study suggests that physical association of PDK1 with Akt1 is sufficient for Akt phosphorylation in the T-loop, which is independent of PIP_3_/PIP_2_ induced plasma membrane translocation [66]. Raptor is a cofactor in the mTORC1 complex without enzymatic activity, but studies suggest that it modulates mTORC1 activity and downstream signaling consequent to its direct/indirect phosphorylation by ERK1, ERK1/2 [67], AMP-activated protein kinase [68], and RSK [69], respectively. Raptor may possibly modulate mTORC1 activity and downstream signaling by inducing conformational changes in mTORC1 and its interacting partners. Thus it would be reasonable to deduce that interaction of Raptor and PDK1 modulates T-loop phosphorylation of Akt1. These studies suggest that targeting Raptor may offer a promising approach for cancer therapeutics. A schematic representation of PDK1/Raptor-mediated phosphorylation of Akt is shown in Figure 6.

The article "Activated α2-Macroglobulin Binding to Cell Surface GRP78 Induces T-Loop Phosphorylation of Akt1 by PDK1 in Association with Raptor" was retracted in 2025. Reasons: duplicated images; overlap with earlier publications; unreliable data; unreliable results or conclusions.

**Figure 6:** A schematic diagram showing the possible mechanism of Raptor-mediated phosphorylation of Akt at Thr^308^ by PDK1.
